# Analysis of the Curative Effect of Continuous Nursing Based on Data Mining on Patients with Liver Tumors

This article has been retracted.

**DOI:** 10.1155/2022/5115089

**Published:** 2022-02-14

**Authors:** ChunFen Peng, LiHong Bao, JingQiong Wang

**Affiliations:** Cancer Center, Union Hospital, Tongji Medical College, Huazhong University of Science and Technology, Wuhan, Hubei, China

## Abstract

Studies have shown that the physical, psychological, and social problems of liver cancer patients are more serious than those of other cancer patients and their quality of life is significantly reduced. This may be related to the poor treatment effect of patients with advanced liver cancer. Patients often have adverse symptoms such as cancer pain, pleural effusion, and ascites, etc., which have a great impact on patients' psychology and recovery from illness. With the change of the medical model, it has become history to rely solely on drugs to care for patients with advanced liver cancer and comprehensive nursing intervention has become very important. Continuous nursing intervention focuses on individualized and full-hearted care, effectively alleviating patients' anxiety and fear and improving patients' environmental adaptability and psychological defense mechanisms. However, in the field of liver cancer, there is no detailed comparison between the efficacy of continuous nursing and traditional conventional nursing. This article applies the hidden Markov model, starts with medical data mining, and describes the process achieved by the application of this article and the analysis of the results obtained by the two nursing methods, which reflect the difference in curative effect evaluation, and it proves that continuous nursing has more advantages in the curative effect of patients with liver tumors.

## 1. Introduction

Liver cancer is one of the common malignant tumors in humans, and its mortality rate ranks third among the malignant tumors of the digestive system in my country. It is worth noting that the incidence of liver cancer is on the rise all over the world [1]. At present, surgical resection is still the first choice for the treatment of liver cancer, but due to the influence of many factors, a large part of clinical patients should not be treated with radical surgery [2, 3]. For example, most liver cancer patients in my country are accompanied by cirrhosis and the lesions are often multiple; the size, location, poor liver function, extrahepatic metastasis, and body failure of the tumor all provide great difficulty and risk for surgical treatment [4, 5]. Hepatic artery intubation embolization chemotherapy is commonly used for patients with unresectable or no surgical indications in the middle and late stages, followed by radiotherapy, chemotherapy, and traditional Chinese medicine treatment [6]. However, current chemotherapy and radiotherapy cannot achieve the goal of completely killing tumor cells. Two prospective randomized controlled studies conducted in Europe and Asia, respectively, show that interventional therapy for liver cancer can significantly prolong the survival time of patients with disease and it is considered to be the first choice for treatment of advanced liver cancer. Although its short-term effect is obvious, the long-term effect is not ideal due to the abundant blood supply of most liver cancers, the rapid formation of collaterals, and the strong ability of angiogenesis. Although the combined application of chemotherapeutic drugs has achieved significant clinical effects, most patients with liver cancer are weaker. The embolization of the tumor-rich blood vessel while infusing a large amount of chemotherapeutic drugs is a great blow to the body [7]. Therefore, how to relieve the physical and psychological pain of liver cancer patients and improve their quality of life has become a research problem that medical staff pays more and more attention to. In recent years, the continuous nursing model has become a new trend in nursing development. Comprehensive and efficient continuous nursing will have a positive impact on patients, families, hospitals, and the society. The United States has included community-based continuous nursing in-laws and regulations in 2010 and injected a large amount of social financial support. After years of practical discussion, the definition of continuous nursing has not yet reached a complete and concrete consensus [8]. Continuous nursing used to be understood as having a family doctor do continuous treatment and care for the patient. Nowadays, due to the increasingly specialized and multidisciplinary characteristics of medical care, continuous nursing refers to the continuous nursing between different medical care providers and medical institutions, with seamless transfer between them [9]. Continuous nursing can also be understood as the degree of continuity of the relationship between nurses and patients [10]. Nursing continuity has multidimensional characteristics, and different definitions emphasize different aspects of continuity. Some definitions focus on the continuity of information and time, some focus on the continuity of the relationship between doctors and patients, some focus on the continuity of the geographic location, some focus on the continuity between disciplines, and some focus on family nursing. The continuous nursing can be summarized into three categories: continuity of information, continuity of management, and continuity of relationships, that is, using information about the patient's past illnesses to provide appropriate treatment and nursing, implementing a coherent method for the management of the patient's health which can satisfy the changing needs of the patient, and maintaining a continuous therapeutic relationship between the patient and one or more healthcare providers [11]. However, the efficacy evaluation of continuous nursing is not perfect. Clinicians and statisticians have proposed many statistical models. Based on the characteristics of continuous nursing clinical longitudinal diagnosis and treatment data, this article applies the hidden Markov model to make longitudinal analysis of continuous nursing data; compared with the predecessors, the method of continuous nursing efficacy evaluation has been improved.

## 2. Related Work

Liver cancer is one of the common malignant tumors in humans, and its mortality rate ranks third among malignant tumors of the digestive system in my country. It is worth noting that the incidence of liver cancer is on the rise all over the world. At present, surgical resection is still the first choice for the treatment of liver cancer. However, due to the influence of many factors, a large part of patients is not suitable for radical surgical treatment in clinical practice. For example, most liver cancer patients in my country are accompanied by liver cirrhosis and the lesions are often multiple; the size, location, poor liver function, extrahepatic metastasis, and body failure of the tumor all provide great difficulty and risk to surgical treatment. Hepatic artery intubation embolization chemotherapy is commonly used for patients with unresectable or no indications for surgery in the middle and late stages, followed by radiotherapy, chemotherapy, and traditional Chinese medicine treatment. However, current chemotherapy and radiotherapy cannot achieve the goal of completely killing tumor cells [12]. However, the traditional medical treatment model is that once the patient is discharged, it means the end of the treatment and nursing relationship. If the patient wants to obtain information related to rehabilitation, he must go to the hospital for follow-up, which brings great inconvenience to the rehabilitation of patients with chronic diseases [13]. On the other hand, continuous nursing focuses on the treatment relationship, the continuity of nursing services, and the sharing of patient information. Patient care services and rehabilitation not only occur in hospitals or medical institutions but also extend to communities or families outside the hospital. Patient information can be shared among different medical institutions and medical staff, so that the continuity of patient care, treatment, and recovery can be ensured. Therefore, continuous nursing requires the participation and close cooperation of all departments, including hospitals, communities, families, and patients. For improving patients' compliance behaviors, mobilizing the enthusiasm of family members to participate in patient care, and expanding service targets from inpatients to the social support system, it breaks the traditional concept of the boundary between the hospital and the community and can deliver new health information to patients and family members can get accurate feedback from patients. According to the new situation or condition of the patient, the content, method, and health guidance can be adjusted in time to realize the interaction between the nurse and the patient, which will help improve the efficiency of medical care and the realization of the network of social health services [14]. Tian and others advocated the concept of “full contract care” in the hospital. Nursing not only includes inpatients but also extends to families, focusing on the guidance on follow-up visits, medication, and rehabilitation of patients after discharge from the hospital [15, 16]. Deng emphasized that patients with spinal cord injury need not only nursing care during hospitalization but also continuous nursing service guidance after discharge [17]. On the basis of chronic obstructive pulmonary disease, Wang and others proposed a continuous nursing model specifically suitable for patients in the mainland. It is characterized by comprehensiveness, cooperation, continuity, and coordination. This model requires hospital nurses and community nurses to cooperate closely to make patients get continuous nursing services when they return to the community or family [18]. In 2005, Mao and Liu established a “continuous nursing service center” in a medical institution in Guangzhou, which specially selected nursing staff with rich nursing experience and strong language skills to carry out continuous nursing. For discharged patients, the door-to-door service is according to personal needs [19]. Different hospital institutions have different understandings and requirements for continuous nursing according to their own hospital's special circumstances, and there is no fixed model for continuous nursing to follow. From a clinical perspective, Xie and Zeng understood the nursing needs during the perichemotherapy period after gastric cancer surgery and formulated continuous nursing plans. The final results showed that they have advantages in improving patients' bad moods and, at the same time, they can also improve patients' satisfaction with clinical care [20]. The study found that by formulating a personalized continuous nursing plan for patients undergoing coronary intervention and implementing continuous nursing from the hospital to the home, the risk can be effectively reduced, the process of coronary atherosclerosis can be minimized, and it can improve the long-term curative effect of coronary stents [21]. Carrying out continuous nursing intervention for patients can effectively improve the compliance of patients with chronic diseases, improve their self-care and management capabilities, and help improve the mental state and condition of patients. Moreover, continuous nursing may effectively reduce complications, improve the quality of life of patients, reduce hospitalization time and hospitalization rate, and save medical expenses. For patients with liver tumors, there is no systematic study of continuous nursing intervention. On the basis of learning continuous nursing experience at home and abroad, this study specifically formulated a continuous nursing model for intervention of patients with liver tumors. This includes comprehensive health education and health guidance in the hospital, cultivating good self-care ability, establishing electronic nursing records, and formulating discharge plans; use telephone and other contact methods to keep in touch with discharged patients and provide nursing consultation, health guidance, and other measures to ensure the continuity of nursing.

The data mining technology is used to evaluate the curative effect of continuous nursing on patients with liver tumors and to study the feasibility of continuous nursing in the treatment of liver tumors. The hidden Markov model (HMM) is a probabilistic model and a type of intelligent algorithm. It has a solid statistical foundation and an effective training algorithm, so it is widely used to describe sequence data or processes. The HMM was originally described in a series of statistical papers by Leonard Baum and other authors in the second half of the 1960s. One of the first applications of HMM was speech recognition that began in the mid-1970s, Fred Jelinek and the Bakers independently proposed the use of HMM to recognize speech, and the error rate of speech recognition is three times lower than that of artificial intelligence and pattern matching methods [22]. In the second half of the 1980s, HMM began to be applied to the analysis of biological sequences, especially deoxyribonucleic acid (DNA). Since then, they have become ubiquitous in the field of bioinformatics [23]. The HMM method has been successfully applied in many fields, such as machine translation and optical character recognition. HMM also has important applications in the fields of bioinformatics and genomics, such as the prediction of protein coding regions in genome sequences, the modeling of interrelated DNA or protein families, and the prediction of second structural elements from basic structures [24]. Liver tumors have a long course of disease and repeated inflammation. The cycle of continuous nursing is also long. It often takes a long time to understand the characteristics of the outcome of continuous nursing for the entire disease. Moreover, liver cancer presents the characteristics of multistate and multistage processes in the development of the disease, and some influencing factors change with time and the disease state; that is, it has a time-dependent characteristic. Therefore, this article chooses the HMM simulation analysis method in clinical decision analysis, which can simulate the various states of the disease over time, evaluate the risk between these different states in each unit of time, and assign the corresponding utility value which takes a predefined end event as the endpoint to simulate the evolution process of the disease to evaluate the researched problem. It is suitable for the correlation of the risk or probability of occurrence of clinical events over time. It is mostly used for the evaluation of clinical intervention measures, the prediction of disease treatment outcome, and the evaluation of the application value of special therapies [25, 26].

## 3. Method

### 3.1. Evaluation of Continuous Nursing Curative Effect Based on HMM

Applying the HMM to the longitudinal data of continuous nursing of patients with liver tumors is a data mining process. On the diagnosis and treatment data of liver cancer patients in clinical Chinese medicine, apply a model that best meets the characteristics of the data, that is, the hidden Markov model; use the method of comparative research to obtain curative effect evaluation indicators; and make reasonable explanations to enrich the method of continuous nursing curative effect evaluation which has great application value. The doctors of the therapeutic effect evaluation group believe that, from the overall effect, continuous nursing is better than traditional conventional nursing. In order to verify the accuracy and practicability of this conclusion, we have done corresponding research work.

Medical data mining is a product of the combination of computer technology, artificial intelligence, statistics, etc. with modern medical care. It has broad application prospects. The method described in this article belongs to medical data mining, which combines computer technology with continuous nursing. The continuous nursing efficacy evaluation was carried out from the medical data, mining methods and rules. Due to the particularity and complexity of medical information itself, compared with conventional data mining, medical data mining has a wide range of objects; the efficiency and robustness of mining algorithms and the accuracy of providing knowledge or decision-making have higher requirements. Medical data mining is an emerging crossdiscipline involving a wide range of technical difficulties. It requires the cooperation of scientific researchers and medical workers engaged in intelligent information processing to strive for the fusion of multiattribute medical information and the efficiency and efficiency of mining algorithms. There have been breakthroughs in key technologies such as accuracy. With the development of technology, medical data mining will play a huge role in the diagnosis and treatment of diseases, medical research and teaching, and hospital management. Medical data has the following characteristics: (1) pattern polymorphism: medical information includes pure data (such as physical sign parameters and laboratory test results), signals, images, text, and voice and video information; (2) incompleteness: the objective incompleteness of the disease information and the subjective inaccuracy of the description of the disease have formed the incompleteness of the medical information; (3) timeliness: the waveforms and images of medical testing are functions of time; there is also a part of medical information that records the patient's medical activities at a certain moment; and (4) redundancy: a medical database is a huge data resource, and a large amount of the same or part of the same information is stored in it every day. The abovementioned characteristics determine the particularity of medical data mining. Due to the characteristics of medical data, the following key problems exist in medical data mining: (1) data preprocessing: the medical database contains a large amount of original information from different sources, which contains a large amount of vague, incomplete, noisy, and redundant information. Before data mining, this information must be cleaned and filtered to ensure data consistency and certainty; (2) information fusion technology: medical information is composed of text, data, waveform signals, images, and a small amount of voice and video signals. These medical data with different physical attributes should be processed with different technologies and measures, and then, the results of the processing should be integrated; (3) fast and robust mining algorithm: medical databases involve a wide range and a large amount of information. To extract knowledge from such a huge database, it takes more time than other databases. Therefore, the efficiency of medical data mining must be considered. At the same time, there are many types of medical databases, and they are dynamically changing, which requires the mining algorithm to have a certain degree of fault tolerance and robustness; and (4) provide accuracy and reliability of knowledge: the main purpose of medical data mining is to provide scientific decision-making for medical activities and management. Therefore, it is necessary to ensure that the knowledge provided by the mining algorithm has high accuracy and reliability. Improving the scientificity and accuracy of mining results is the key to whether medical data mining can be applied in practice.

### 3.2. Overview of the Program Flow

The preprocessed data is read from the symptom table of the database according to the specified input format and stored in a plain text file to lay the foundation for the following learning process. First, use the improved “segmental *k*_means” algorithm to cluster the observation vectors stored in the text file, and then, learn the initial model parameters, that is, determine the “initHMM.” Secondly, use the classic “Baum_Welch” algorithm in the HMM to learn the model parameters of “initHMM” multiple iterations and calculate the Kullback-Leibler divergence (KL) distance between the new iteration model and the previous iteration model multiple times, and the KL distance for each iteration both will decrease, indicating that the iteration is closer to the real model. After iterative convergence, the final “learntHMM” model parameters are obtained. We can compare and analyze the model parameters, assign actual meaning to each state, and analyze the transition probability in the state transition probability matrix. After that, it enters the testing phase. According to the final iterative “learntHMM” model, test vectors are randomly generated. The improved forward and backward algorithm of the hidden Markov model can calculate the probability of each test sequence. The Tebi algorithm calculates the state sequence that this observation vector is most likely to correspond to under this model. The specific flow chart is shown in Figure 1.

### 3.3. Implementation of Related Algorithms

#### 3.3.1. Multiple Observation Sequence Training

In actual use, more than one observation sequence is often used to train an HMM. Then, when training the HMM with *N* observation sequences, the reevaluation formula of the “Baum_Welch” algorithm must be modified. Let *N* observation sequences be *L*^(*n*)^, *n* = 1, 2, ⋯, *N*, where *L*^(*n*)^ = *l*_1_^(*n*)^, *l*_2_^(*n*)^, ⋯, *l*_*T*_*n*__^(*n*)^, assuming that each observation sequence is independent, at this time:

(1) $$\begin{array}{c} F\left(L\;|\;\mu \right)=\overset{N}{\underset{n=1}{\prod }}F\left(L^{\left(n\right)}\;|\;\mu \right). \end{array}$$

Since the reevaluation formula is based on the frequency of occurrence of different events, for *N* training sequences, the reevaluation formula is revised to

(2) $$\begin{array}{c} {\bar{\omega }}_{i}=\overset{N}{\underset{n=1}{\sum }}\gamma_{t}^{\left(n\right)}\delta_{t}^{\left(n\right)}\;|\;F\left(L^{\left(n\right)}\;|\;\mu \right),\\ {\bar{p}}_{ij}=\frac{\sum_{n=1}^{N}\sum_{t=1}^{T_{n}-1}\gamma_{t}^{\left(n\right)}\left(i\right)p_{ij}q_{j}\left(l_{t+1}^{\left(n\right)}\right)\delta_{t+1}^{\left(n\right)}\left(j\right)\;|\;F\left(L^{\left(n\right)}\;|\;\mu \right)}{\sum_{n=1}^{T}\sum_{t=1}^{T_{n}-1}\gamma_{t}^{\left(n\right)}\left(i\right)\delta_{t}^{\left(n\right)}\left(j\right)\;|\;F\left(L^{\left(n\right)}\;|\;\mu \right)},\;1\leq i,j\leq A, \end{array}$$

where *p*_*ij*_ is a matrix with the *A* row and *A* column.

(3) $$\begin{array}{c} {\bar{q}}_{jk}=\frac{\sum_{n=1}^{N}\sum_{t=1,o_{t}=V_{k}}^{T_{n}}\gamma_{t}^{\left(n\right)}\left(j\right)\delta_{t}^{\left(n\right)}\left(k\right)\;|\;F\left(L^{\left(n\right)}\;|\;\mu \right)}{\sum_{n=1}^{N}\sum_{t=1}^{T_{n}}\gamma_{t}^{\left(n\right)}\left(j\right)\delta_{t}^{\left(n\right)}\left(k\right)\;|\;F\left(L^{\left(\text{n}\right)}\;|\;\mu \right)},\;1\leq j\leq A,1\leq k\leq B, \end{array}$$

where *q*_*ij*_ is a matrix with the *B* row and *B* column.

#### 3.3.2. Data Underflow Problem

In the forward and backward algorithm and the “Baum_Welch” algorithm, there are recursive calculations of *γ*_*t*_(*i*) and *δ*_*t*_(*i*). Since all the quantities are less than 1, as *t* increases, *γ*_*t*_(*i*) will rapidly tend to 0 and *δ*_*t*_(*i*) will tend to 0 as *t* decreases. In order to solve this data underflow problem, the method of increasing the scale factor can usually be adopted to modify the relevant algorithm. The processing process is as follows: (1) processing of *γ*_*t*_(*i*):

(4) $$\begin{array}{c} \gamma_{n}\left(i\right)=\omega_{i}q_{i}\left(l_{n}\right),\;1\leq i\leq A,\\ \gamma_{n}^{*}\left(i\right)=\frac{\gamma_{n}\left(i\right)}{\sum_{i=1}^{A}\gamma_{n}\left(i\right)}=\frac{\gamma_{n}\left(i\right)}{\varphi_{n}},\;1\leq i\leq A,\\ {\tilde{\gamma }}_{t+1}\left(j\right)=\left[\overset{A}{\underset{i=1}{\sum }}\gamma_{n}^{*}\left(i\right)p_{ij}\right]q_{j}\left(l_{t+1}\right),\;1\leq j\leq A,t=1,2,\cdots ,T-1,\\ \gamma_{t+1}^{*}\left(\text{j}\right)=\frac{{\tilde{\gamma }}_{t+1}\left(j\right)}{\sum_{j=1}^{A}{\tilde{\gamma }}_{t+1}\left(j\right)}=\frac{{\tilde{\gamma }}_{t+1}\left(j\right)}{\varphi_{t+1}},\;1\leq j\leq A,t=1,2,\cdots ,T-1, \end{array}$$

where $\varphi_{t+1}=\sum_{j=1}^{A}{\tilde{\gamma }}_{t+1}\left(j\right)$ and (2) processing of *δ*_*t*_(*i*):

(5) $$\begin{array}{c} \delta_{T}\left(i\right)=1,\;1\leq i\leq A,\\ \delta_{T}^{*}\left(i\right)=1,\;1\leq i\leq A,\\ {\tilde{\delta }}_{t}\left(i\right)=\overset{A}{\underset{j=1}{\sum }}p_{ij}q_{j}\left(l_{t+1}\right)\delta_{t+1\;}^{*},\;1\leq i\leq A,t=T-1,\cdots ,1. \end{array}$$

When adjusting *δ*_*t*_(*i*), the scale factor used is the same as when adjusting *γ*_*t*_(*i*). The main consideration is that the value ranges of *δ*_*t*_(*i*) and *γ*_*t*_(*i*) are comparable, and the value of *δ*_*t*_(*i*) can be adjusted to a suitable range through the same scale factor.

#### 3.3.3. KL Distance

From the perspective of probability measurement, Rabiner and Juang proposed to measure the similarity between two hidden Markov models *ρ*_1_ = {*ω*_1_, *C*_1_, *D*_1_} and *ρ*_2_ = {*ω*_2_, *C*_2_, *D*_2_}. Assuming that *ρ* produces a set of *K* feature vectors {*L*^(*k*)^ | 1 ≤ *k* ≤ *K*}, then, the similarity measure between *ρ*_1_ and *ρ*_2_ is defined as

(6) $$\begin{array}{c} R\left(\rho_{1},\rho_{2}\right)=\underset{K⟶\infty }{\lim}\frac{1}{K}\overset{K}{\underset{k=1}{\sum }}\left\{\log F_{{L_{1}}^{\left(k\right)}}\left[\rho_{1}\right]-\log F_{{L_{1}}^{\left(k\right)}}\left[\rho_{2}\right]\right\}, \end{array}$$

where *F*_*L*^(*k*)^_[*ρ*] represents the probability of model *ρ* generating a feature vector *L*^(*k*)^. Obviously, the smaller the *R*(*ρ*_1_, *ρ*_2_), the greater the similarity between the two. In the actual calculation, each *L*_1_^(*k*)^ can be obtained from *ρ*_1_ by the Monte Carlo method. As long as the value of *K* is large enough, a sufficiently accurate result can be obtained. Equation (6) is not a symmetry measure, and you can use equation (6) to construct a symmetry measure:

(7) $$\begin{array}{c} R_{s}\left(\rho_{1},\rho_{2}\right)=\frac{1}{2}\left\{R\left(\rho_{1},\rho_{2}\right)+R\left(\rho_{2},\rho_{1}\right)\right\}. \end{array}$$

Simulation experiments on the distance measurement show that the difference between the parameters *ω* and *C* has a much smaller effect on the distance *R* than the difference between the parameter *D* and the distance.

#### 3.3.4. Segmental *k*_Means Algorithm

The classic clustering technique is called *k*-means. First, specify the number of clusters to be found, which is the parameter *k*. Then, randomly select *k* points as the center of the cluster. According to the common Euclidean distance measurement, all the instances are assigned to their nearest cluster centers. The next step is to calculate the centroid, or average, of each cluster where the instance is located. This is the “mean” part. Finally, repeat the whole process with a new cluster center. The iteration process continues until in successive rounds, and the points assigned to each cluster are the same as the points assigned in the previous round. At this time, the center of the cluster is already fixed, and it will always remain. This clustering method is simple and effective, and it is easy to prove that the centroid is selected as the center of the cluster, so that the sum of the squares of the distance from each point in the cluster to the center is minimized. In the late 1980s, the segmental *k*_means algorithm was proposed and widely adopted. Its basic idea is to continuously adjust the parameters of the HMM according to the current maximum likelihood state sequence until the template converges. Although the HMM parameter reestimation formula used in this algorithm is simple and clear, because this algorithm does not take the detection rate as the objective function, the HMM obtained by training is relative to the overall performance of the detection system. The language is not the best. Secondly, when implementing this algorithm, it is difficult to determine the threshold for judging whether the template has converged. This is mainly due to the inconsistency of the symptoms and characteristics of the training content itself. Therefore, I have made some improvements to ensure the robustness of the program.

## 4. Experiment and Analysis

### 4.1. Normative Organization of Data

How to organize and standardize experimental data requires not only corresponding data cleaning but also data merging. The work of data cleaning and data merging can be performed on the existing extraction-transformation-loading (ETL) platform. After removing the singular values from the data, we need to further process the data. In order to prove the researcher's work hypothesis, the experimental group research needs to design an observation group. Comparative research is an important method of clinical trials. It explains the efficacy and safety of a therapy, and a control group must be set up. The control group is a group of subjects under the same conditions as the experimental group. The only difference is that the experimental group receives continuous nursing while the control group receives traditional routine nursing. The purpose of setting up a control group is to determine whether the subjects' changes before and after nursing are caused by continuous nursing, rather than other reasons. Clinical trials require that the test group and the control group come from the same population of subjects. Not only at the beginning of the experiment, the basic conditions of the two groups of subjects are corresponding or similar, but during the experiment, except for the different care methods of the experiment, other conditions must be consistent. If the conditions of the two groups of patients are inconsistent, it will affect the analysis and interpretation of the results, and the estimated treatment effect will deviate from the true effect value. Therefore, when we are doing data preprocessing, under the guidance of clinicians and professional nurses, all patient data are strictly and reasonably divided into traditional routine care and continuous nursing groups according to the content of care. Except for different nursing care, the two groups of patients maintained the same conditions and met all the requirements of clinical trials for comparative research. Such grouped data for efficacy evaluation has laid a solid foundation for the rationality of the results.

### 4.2. Analysis of Experimental Results

The therapeutic effect evaluation believes that continuous nursing is better than traditional conventional nursing from the overall effect. Combining the continuous nursing curative effect evaluation and the HMM discussed in this article, we realize that the state transition matrix of the HMM can objectively reflect the curative effect evaluation from a certain aspect. The specific process of efficacy was evaluated by the state transition matrix. First, we show the vector composed of three symptoms: pain, fatigue, and nausea and vomiting. It is divided into the traditional routine nursing group and the continuous nursing group. In the application program, we constructed the result of running on. In order to facilitate comparison, without involving specific clinical implications, we divide the two sets of data into three states: light, medium, and heavy; see Tables 1 and 2 and Figures 2 and 3 for details.

After correlating the status with the clinical condition, we can proceed to the link of efficacy evaluation. A key indicator of efficacy evaluation is the rate of improvement. In layman's terms, it is the probability of transition from a state of heavy to a moderate state, or even to a light state, that is, the probability of a patient's transition from a more severe state to a remission state or the percentage of patients whose symptoms have alleviated. It is not difficult to draw the following results from the above analysis results: (1) shift from symptoms to mild symptoms: 0.5 for the traditional routine care group and 0.95 for the continuous nursing group. This shows that in the process of transitioning from the state to the light state, the effect of the continuous nursing group is much better than that of the traditional conventional nursing group; (2) from severe symptoms to mild symptoms: the metastasis probability of the traditional conventional care group is 0.15, while that of the continuous nursing group is 0.2, which shows that severe liver cancer has a certain effect on both types of care, while the performance of the continuous nursing group is more prominent; and (3) from severe symptoms to symptoms: the transition probability of the traditional routine care group is 0.75, while the probability of the continuous nursing group is 0.9. The difference between the two groups is not very big, but the continuous nursing group has a slight advantage.

The data analyzed above is for our preliminary data mining, and only three symptoms are taken, namely, pain, fatigue, nausea, and vomiting. However, these three symptoms are not enough to reflect the changes in the condition of liver cancer patients, or from a clinical point of view, these three symptoms are not universal in simulating the development process of the disease. Therefore, in the following analysis, we have selected the best reflection of the condition of liver cancer. The symptoms developed are the following 10 symptoms extracted from the Oracle data warehouse: pain, fatigue, nausea and vomiting, fever, abdominal distension, ascites, cough, shortness of breath, loss of appetite, and gastrointestinal reactions. In other words, in the input file processed by the model, each vector is 10 dimensional, and there are 2 to 30 vectors in a diagnosis and treatment behavior of each patient, depending on what each patient does in each admission. The number of physical examinations and items the traditional routine nursing group has 180 diagnosis and treatment behaviors, and the continuous nursing group has 360 diagnosis and treatment behaviors. We used the learning process of this huge dataset to evaluate the efficacy and found that the state transition probability of 10 symptoms learned is different from the transition probability of 3 symptoms.  Table 3 is the symptom score table of the hidden Markov model learned by the traditional routine care group.

Table 4 is the symptom score table of the hidden Markov model learned by the continuous nursing group.

Figure 4 is the average symptom score of different symptoms under the two nursing groups.

The two nursing groups compared the mean values and found that among the three corresponding symptoms, the mean symptom mean value of continuous nursing was lower than the mean symptom mean value of traditional conventional nursing. Combined with our initial assignment of symptoms, it shows that in each state, the actual condition of patients in continuous nursing is better than that of patients in traditional routine care.

Figures 5–7 show the state transition probability of traditional conventional nursing and continuous nursing. S1, S2, and S3 all represent different pathological features of liver cancer.

It can be seen that even if the 10 common symptoms of liver tumors are selected, the performance of continuous nursing is still stronger than traditional conventional nursing.

## 5. Discussion

The incidence of liver cancer in my country has been increasing at an annual rate of over 10% in the past 20 years, and it has become one of the most common clinical malignancies [27]. In recent years, the expertise and advantages of professional nursing in the prevention and treatment of liver cancer have attracted worldwide attention, especially in improving symptoms, improving the quality of life, and prolonging survival [28]. In the clinical treatment of liver cancer patients, interventional therapy has the advantages of small trauma and significant efficacy for advanced patients and has become one of the main treatment methods adopted in the clinic. However, the patient's postoperative hospital stay is short, the physiological function is significantly reduced, and the mood fluctuations are relatively large, so it is still necessary to carry out the necessary nursing intervention for the patient after discharge [29, 30]. The continuous nursing mode can effectively improve the postoperative quality of life of patients with early primary liver cancer, improve self-care ability, achieve a more ideal nursing effect, and further improve the rehabilitation effect of advanced liver cancer patients after interventional treatment, which is of great clinical significance. Through literature study and personal practice, we have realized that nursing has a good effect on the treatment of liver cancer. The evaluation of nursing curative effect is a very comprehensive and very complex subject, which not only involves the theoretical level and the way of thinking but also is closely related to the methodology and practical operation. The scientific and objective evaluation of the characteristics of continuous nursing in the treatment of liver cancer is of inestimable value for expanding the application fields of professional nursing and promoting the academic development of nursing. The data derived from the actual nursing process is observational data, which is a large-scale dataset with unequal time intervals and missing response indicators. It is very difficult to use the longitudinal analysis method of the existing statistical analysis software to conduct research. Continuous care as a new mode of care can understand the progression of the patient's condition, while implementing some community care for the patient and regular return visits [31]. Not only does it improve the patient's emotional condition, optimize their quality of life, and improve the patient's ability to care but it also improves the quality of care and satisfaction which is very beneficial to the patient's treatment outcome and has been confirmed in many studies [32, 33]. This article uses the HMM to carry out the longitudinal analysis of continuous nursing and evaluates the efficacy of the traditional conventional nursing and continuous nursing methods of liver cancer nursing data. The difference between the two methods is found, and the HMM is verified. The effect of the husband model in the evaluation of medical efficacy.The data in this article uses the clinical data of 1000 cases of liver cancer in an industry special project of the Chinese Medicine Administration for analysis and research. After data cleaning and irregular data removal, the dataset includes 400 cases of traditional routine nursing and 400 cases of continuous nursing. This paper trains the HMM through the dataset, obtains the transition probability in the model, uses the improvement rate learned from the model to evaluate the curative effect, and objectively demonstrates the difference between the two nursing methods.

## 6. Conclusion

The experimental results show that the use of HMM for the longitudinal analysis of nursing data is effective.

## Figures and Tables

**Figure 1:** The process of learning and testing with HMM.

**Figure 2:** The state of different symptoms under traditional routine nursing.

**Figure 3:** The state of different symptoms under continuous nursing.

**Figure 4:** Average symptom score of different symptoms in two nursing groups.

**Figure 5:** State transition probability of different nursing methods in the mild state.

**Figure 6:** State transition probability of different nursing methods in the moderate state.

**Figure 7:** State transition probability of different nursing methods in the severe state.

**Table 1:** Transition probability in different states under routine nursing.

State	Mild			Moderate			Severe		
Transition probability	0.01	0.15	0.01	0.5	0.05	1	0.15	0.75	0.1

**Table 2:** Transition probability in different states under continuous nursing.

State	Mild			Moderate			Severe		
Transition probability	0.09	1	0	0.95	0	0.01	0.2	0.9	0.99

**Table 3:** Symptom scores in different states under traditional routine care.

Mean	1	2	3	4	5	6	7	8	9	10
Mild	12.5	12.0	11.2	11.4	20.5	20.6	12.8	10.5	15.5	13.0
Moderate	13.6	14.4	12.5	12.6	18.4	16.2	18.8	26.5	30.3	8.7
Severe	18.2	15.4	10.5	13.7	32.5	24.6	21.5	27.5	16.8	13.3

**Table 4:** Symptom scores in different states under continuous nursing.

Mean	1	2	3	4	5	6	7	8	9	10
Mild	11.2	9.6	10.7	10.4	16.5	18.2	11.2	11.5	13.4	14.3
Moderate	12.5	10.4	9.5	10.6	15.4	17.2	16.8	23.6	24.5	16.5
Severe	16.2	12.4	8.5	10.7	26.5	24.6	21.8	25.3	18.8	14.2

## Data Availability

No data were used to support this study.
